# Artificial Intelligence-Based Recommendation and Application of Public Services in Smart Cities

This article has been retracted.

**DOI:** 10.1155/2022/8958865

**Published:** 2022-08-30

**Authors:** Jin Zhou

**Affiliations:** ^1^School of Public Administration, Sichuan University, Chengdu 610065, China; ^2^Hubei Minzu University Library, Hubei, En'shi 445000, China

## Abstract

With the promotion and application of information technology, smart cities based on artificial intelligence have become the best choice for the government to solve urban problems, connect urban citizens, and provide quality public services. From the initial information city and digital city to the current smart city, the construction of smart cities has undergone profound changes with five major characteristics: big data, intelligence, innovation, interaction, and integration, and Internet giants have emerged in the field of public services in smart cities. Internet giants are emerging in the construction of public service platforms for smart cities, and traditional smart city construction enterprises are also expanding various forms of urban operation services through the form of “Internet+“. Nevertheless, there is still a gap between the quantity and quality of China's smart cities compared with developed countries, and there is a need to build a number of pilot smart cities characterized by the linkage of artificial intelligence technology and public services, easy to promote, and sustainable development. The smart city construction model with public services as the core has research value and has the possibility of becoming the mainstream development in the future. Therefore, exploring the organic combination of AI technology and urban public services is the key to answer whether AI technology can promote the improvement of urban public services.

## 1. Introduction

China's urbanization process is accelerating, the level of economic development is rapidly increasing, the urban population is constantly coming in and expanding, and residents' requirements for daily life and public services are also increasing [1]. Under such circumstances, the traditional public service model is increasingly unable to adapt to these changes [2]. In the face of the growing population size and the increasing requirements for living experience, the contradiction between insufficient urban carrying capacity and low level of public services has forced the need for rapid transformation in the construction of urban public service facilities. Smart cities are undoubtedly a powerful means to break this bottleneck [3]. SmartCity is an intelligent self-awareness, self-adaptation, and self-optimization based on comprehensive perception and interconnection of ubiquitous information using new-generation information technology to achieve seamless connection and cooperative linkage among people, things, and urban functional systems, so as to make intelligent responses to urban service demands, such as people's livelihood, environmental protection, public safety, urban functions and business activities, and form a safe, convenient, efficient, and green city with sustainable endogenous power. It can form a safe, convenient, efficient, and green city form with sustainable endogenous power [4]. It can make the services and facilities in the city make intelligent and rapid responses to better perform their functions and guarantee the development of people's livelihood [5]. Public service facilities, which are the concrete manifestation of the city's services for its residents, are the means of expression of all aspects of the city's functions [6]. Whether they are truly organically combined with modern information means, scientific planning and innovation, and ultimately meet the requirements of intelligent services, is the biggest criterion to measure whether a smart city is truly built.

For the construction of urban public service facilities, the main issues to be considered are the rational allocation of space and the correspondence between functions and needs, so when using the theory of smart cities for construction, these issues should also be considered, and on this basis, a more “intelligent” model and thinking should be used to deal with problems, introduce new technologies, and bring wisdom into play [7]. After setting this basic direction, it is necessary to consider various factors, such as input, efficiency, effectiveness and balance. For example, when planning the space, it is necessary to ensure the maximum representation of functions, but also to take care not to take resources from other areas and to ensure the overall coordination and science of urban planning. When designing the specific locations and configurations of various service facilities, the degree of residents' demand for different services should be actually investigated so that the response speed and priority of the service facilities meet the actual needs, such as appropriately increasing the number and density of some services with high pedestrian flow and urgent demand [8]. In addition, when designing and planning, it is also necessary to apply a developmental perspective as much as possible and introduce innovative means and technologies so that traditional public service facilities can be infused with new vitality, keep up with the times, and strive to meet the gradually growing individualized needs of residents. In this way, it is also expected to enhance the residents' sense of identity and life experience in the city, pull the development of the city, and improve the overall development level and comprehensive strength of the city.

The construction of smart cities is also inseparable from the application of big data. Through data collection and macro analysis of city residents, we can summarize the demand and intensity of various public service facilities and residents' tendency to choose them to help make more reasonable planning and settings [9]. By applying various perception-based technologies and location identification systems to draw precise point-to-point planning maps and incorporate detailed information of residents in real time, we can gain a deeper and more comprehensive understanding of residents' daily needs and living habits and improve the efficiency of public service facilities in a targeted manner.

At present, the construction and development of smart cities suffer from the lack of regional characteristics, insufficient development planning, unbalanced construction and application, imitation over R&D, and difficulty in integrating resources, while the research on smart cities emphasizes technology over application, the disconnection between high-tech and application services, and the deviation between concept and practice. How to plan urban public service facilities scientifically and effectively, and how to apply wisdom technology to public services in combination with social needs are the key points and difficulties of smart city construction, which is also the main theme of this paper.

## 2. Related Work

Since the theory of “smart city” was proposed, it has been discussed and analyzed by various parties, and the theoretical system is becoming more and more enriched and mature, and the basic connotation is changing [10, 11]. At present, the discussions and concerns about smart cities are mainly focused on the technical level and the policy level: at the technical level, the concern is about the technology to be introduced and its feasibility; at the policy level, the discussion is about the government's attitude and guidance, and the presence of democratic forces is considered [12]. In addition, many scholars in China have been committed to constructing and filling the basic framework of smart city theory, trying to explore deeper connotations, combining local characteristics or even local features, and constructing a comprehensive and detailed theory from which all places can learn and form a system that truly fits our national conditions [13].

Technology has always been the focus of attention, and although the combination of information technology and urban construction is not a new concept, how to use it skillfully and rationally needs to be explored in depth [14]. At present, smart cities are applied to a variety of technical means, of which the supporting technologies mainly include cloud computing, information collection and integration, artificial intelligence identification, etc. And with the continuous development of information technology and frequent results, more new technologies are bound to be applied to the construction of smart cities [15]. At present, several cities in China have incorporated the construction of smart cities into their development plans, and the applicable technologies will be different for these cities with different development directions and human geographic connotations [16]. How to use the technology comprehensively according to their own characteristics and realize the maximum value of the technology is also a problem that needs to be faced directly [17].

The smooth construction and development of smart cities cannot be achieved without the support and guidance of policies [18]. In this regard, relevant departments and experts have studied and discussed the policies. Smart cities involve economy, people's livelihood, humanities, environment, etc., which cannot be favored over others, otherwise, it will easily cause unbalanced and unstable conditions, which is the reason why policy forces are needed to intervene. The policy research should start from the position of each resident, close to the people's life, and try to achieve real benefit to the people.

In the context of artificial intelligence, it is of great importance how to better recommend and apply public services in smart cities, in which effective intelligent recommendation algorithms are necessarily needed. The basic idea of recommendation system, as a tool to facilitate people to quickly and accurately locate the items they are interested in among a large number of item choices in the era of big data, is to extract the characteristics of users and items from their historical data by building a model, and to recommend items to users in a targeted manner using the trained model [19]. Research on applying reinforcement learning to recommender systems has received increasing attention. The first exploratory model that applies deep reinforcement learning to recommender systems is DRN [20], which constructs a basic framework for recommender systems, and the block diagram is shown in Figure 1.

In such a reinforcement learning framework, the learning process of the model can be iterated continuously, and the iterative process has the following main steps.

1. Initialize the recommendation system (intelligent body)
2. The recommendation system performs news ranking (action) based on the current collected data (state) and pushes it to the website or app (environment)
3. The user receives a list of recommendations and clicks or ignores (feedback) a recommendation result
4. The recommendation system receives the feedback and updates the current state or updates the model-by-model training
5. Repeat step 2

There have been many research results about deep reinforcement learning-based recommender systems, such as the literature [21] and others applied DQN to social networks. Applied DQN to a trust recommendation system based on social networks, applied to an intelligent body to learn the dynamic representation of trust between users and recommend users based on that trust value; literature [22] applied DDQN to recommendation suggestions, solving the problems of low recommendation accuracy, slow speed, and cold start; literature [23] applied DDPG algorithm to stored recommendations, solving the problem of sparse user data. The literature [24] applied the Actor-Critic algorithm to list-based recommendation, solving the problem that the traditional recommendation model can only model the recommendation process as a static process. The above research results and the numerous studies not listed above use the nature of reinforcement learning itself to solve the recommendation problem, and rarely consider the problem from the recommendation perspective.

## 3. Practical Scheme

By dividing the basic public service items, the dimensions of measuring the level of public services in smart cities were classified as public education (PE), social security (SC), medical health (MHC), housing security (HC), public culture (PC), and social services (SS). The smart city pilot started in 2013, so the panel data of 31 provinces (regions and cities) in China from 2014 to 2018 were selected for the empirical study. The data were obtained from China Statistical Yearbook, China Science and Technology Statistical Yearbook, and National Housing Fund Report from 2014 to 2018. In order to exclude the influence of factors, such as interaction terms and reveal the relationship between AI technology and public service level, control factors are added and a panel data model is constructed:

(1) $$\begin{array}{c} PE_{ti}=\alpha_{0}+\beta_{1}DI_{ti}+\beta_{2}DO_{ti}+\beta_{3}GDP_{ti}+\beta_{4}FDI_{ti}+\beta_{5}INF_{ti}+\beta_{6}PS_{ti}+\epsilon_{ti}\text{,}\\ SC_{ti}=\alpha_{0}+\beta_{1}DI_{ti}+\beta_{2}DO_{ti}+\beta_{3}GDP_{ti}+\beta_{4}FDI_{ti}+\beta_{5}INF_{ti}+\beta_{6}PS_{ti}+\epsilon_{ti}\text{,}\\ MHC_{ti}=\alpha_{0}+\beta_{1}DI_{ti}+\beta_{2}DO_{ti}+\beta_{3}GDP_{ti}+\beta_{4}FDI_{ti}+\beta_{5}INF_{ti}+\beta_{6}PS_{ti}+\epsilon_{ti}\text{,}\\ HC_{ti}=\alpha_{0}+\beta_{1}DI_{ti}+\beta_{2}DO_{ti}+\beta_{3}GDP_{ti}+\beta_{4}FDI_{ti}+\beta_{5}INF_{ti}+\beta_{6}PS_{ti}+\epsilon_{ti}\text{,}\\ PC_{ti}=\alpha_{0}+\beta_{1}DI_{ti}+\beta_{2}DO_{ti}+\beta_{3}GDP_{ti}+\beta_{4}FDI_{ti}+\beta_{5}INF_{ti}+\beta_{6}PS_{ti}+\epsilon_{ti}\text{,}\\ \frac{1}{n}\overset{n}{\underset{i=1}{\sum }}\text{Ave}\_{\text{Reward}}_{i},n\text{,} \end{array}$$

where *PE*_*ti*_ denotes the level of public education in city *i* (*i*  = 1, 2,…, *n*) in year *t*, *SC*_*ti*_ denotes the level of social security in city *i* in year *t*, *MHC*_*ti*_ denotes the level of health care in city *i* in year *t*, *HC*_*ti*_ denotes the level of housing security in city *i* in year *t*, *PC*_*ti*_ denotes the level of public culture in city *i* in year *t*, *SS*_*ti*_ denotes the level of social services in city *i* in year *t*, *DI*_*ti*_ denotes the AI technology input of city *i* in year *t*, *DO*_*ti*_ denotes the AI technology output of city *i* in year *t*, *GDP*_*ti*_ denotes the economic level of city *i* in year *t*, *FDI*_*ti*_ denotes the openness level of city *i* in year *t*, *INF*_*ti*_ denotes the infrastructure level of city *i* in year *t*, *PS*_*ti*_ denotes the population size of city *i* in year *t*, and *ϵ*_*ti*_ is a random disturbance term.

Public education (PE) is measured by the pupil–teacher ratio in elementary schools. With the popularization of quality education, the teacher–student ratio has become an important criterion for the improvement of educational strength. Social Security (SC) is measured by the urban registered unemployment rate. With the development of the economy, the role of unemployment insurance in preventing unemployment and promoting employment is becoming more and more important, and has become a booster and safety valve for economic development and social stability. Medical Health Care (MHC) is measured by the number of beds in medical and health institutions per 1,000 people. With the development of modern economy, the residents' demand for medical and health resources allocation is getting higher and higher, and the number of medical and health institution beds in a region represents the intensity of medical and health security in that region. Housing security (HC) is measured by the amount of CPF contributions. The value-added income of the CPF provides a source of funds for the construction of low-cost housing and supports low-income families in solving their housing problems, reflecting the special function of housing security. Public culture (PC) is measured by the number of books per capita in public libraries. In terms of equalization, standardization, digitalization, and socialization, libraries have always led the development of public cultural services. Social services (SS) are measured by the number of elderly beds per 1,000 elderly people. “The 13th Five-Year Plan points out that the number of social service beds for the elderly can be used as the basis for judging the assistance and welfare subsidies for the elderly.

Artificial intelligence investments are based on trading logic and mathematical models given to computers by computer programmers. Computers are programmed to capture investment opportunities across the market and put them into practice, and all trading moves are made based on models, algorithms, and logic that can overcome human weaknesses, such as greed, fear, and fluke. Investment in artificial intelligence (DI) is measured by the intensity of investment in research and experimental development (R&D) in each region. Capital is the blood of innovation activities and is an important link to continuously support the development of innovation in the digital economy. R&D investment intensity can better measure the R&D capital investment in digital information technology. Artificial intelligence technology output (DO) is measured by the number of patent applications per 10,000 people in each region. Patent data can better reflect technological innovation and better demonstrate the level of AI technology in cities.

Economic level (GDP), measured by per capita gross regional product; openness level (FDI), measured by foreign fixed asset investment; infrastructure (INF), measured by per capita urban road area; and population size (PS), measured by the number of population at the end of each year, are given in Tables 1–3.

This section introduces the proposed model for Smart City Recommendation (SCR), which uses user interests as the states seen by the intelligences in deep reinforcement learning as a way to accomplish the intelligent recommendation task. To capture the long-term interest of users, this paper uses a long- and short-term memory network (LSTM) with state enhancement units to learn the browsing records of users over a longer period of time, and retention ratios in the network through three gating units.

We use the attention mechanism as the base model for extracting users' short-term interests. It is assumed that the user's short-term interest can be extracted from three consecutive browsing records (item1, item2, and item3), which are coded to form vector *γ*. After that, the three vectors are calculated as respective Queries vector, Keys vector, and Values vector according to different parameters *W*_*Qi*_, *W*_*Ki*_, *W*_*Vi*_(*i*=1,2,3) and combined into a matrix form, and then the following formula is used to calculate the self-attentive value of each record is calculated by the following formula.

(2) $$\begin{array}{c} Z*=\text{softmax}\left(\frac{Q\times K^{T}}{\sqrt{d_{k}}}\right)\text{,} \end{array}$$

where *Q*, *K*, *V* are the matrices based on *X*_1_, *X*_2_, *X*_3_ vectors combined as Queries vector, Keys vector, and Values vector, respectively, and *d*_*k*_ is the length of a browsing record. *Z* ^*∗*^ is the matrix of the final calculated vector of short-term interests of the user reflected by each item.

The final short-term interest of the user is achieved by directly summing the user short-term interest vectors reflected by each item, i.e.,

(3) $$\begin{array}{c} \text{shortinterest}=Z_{1}+Z_{2}+Z_{3}+\cdots +Z_{n}\text{.} \end{array}$$

The *Z*_*i*_ in the equation represents the user's short-term interest reflected by the *i* th browsing record. *i* has a temporal characteristic, i.e., the larger *i* is, the closer it is to the current moment, and *Z*_*i*_ the closer the interest expressed is to the user's current interest. Careful consideration reveals that when multiple *Z*_*i*_'s are superimposed, the trend of current user short-term interest is diluted as *Z*_*i*_'s are superimposed. To solve this problem, this paper improves short interest by adding weights to the short-term interests expressed by each browsing record in order, and the more backward the time, the greater the weight assigned to the user's short-term interests, as expressed by the formula

(4) $$\begin{array}{c} \text{shortinterest}=\frac{1}{n}Z_{1}+\frac{2}{n}Z_{2}+\frac{3}{n}Z_{3}+\cdots +Z_{n}\text{.} \end{array}$$

The final model is called *T*-self-attention, and the weight of the interest vector in the short-term interest composition is assigned in time sequence. By embedding the long and short-term interest extraction module into the Actor network of the DDPG algorithm, the purpose of updating the parameters of the long- and short-term interest extraction module network while training the Actor network is achieved, and an improvement of the Actor network is shown next. The pseudocode of the algorithm of SCR is given in Algorithm 1.

## 4. Case Study

In order to prove the effectiveness of our scheme, we have experimented and analyzed it on a dataset. In this paper, the following rules are followed in both training and testing phases: the user browsing sequence is denoted as: *S*_*u*_=(*I*_1_, *I*_2_, *I*_3_,…, *I*_|*S*_*u*_|_) , where *I*_*i*_ denotes the *i*-th record of the item viewed by the user. The first 0.8*∗*|*S*_*u*_| of each user's browsing records are used as the training set, and the remaining data are used as the test data. During training, the browsing records in the training set are input into the model in order of users, and for each record, the model predicts the rating of the recommendations contained in the record, and the reward value is calculated based on the difference between the real rating and the predicted rating and fed back to the intelligence, and the algorithm optimizes the model based on the reward value. The operations during testing are similar to those during training, but there is no model optimization operation.

(1)   Action space: in this paper, the original scores are normalized to map the range of values to the interval [0, 1], which becomes (0, 0.25, 0.5, 0.75, 1). Meanwhile, the results are mapped to the [0, 1] interval using the sigmoid activation function at the fully connected layer of the algorithm using the floating-point data with continuity generated each time as the action, i.e., the predicted recommendation scores. Therefore, the action space of this model is a continuous space in the interval of [0, 1].
(2)   State space: the user browsing records are treated as an observation, and the extracted interests are used as states after interest extraction by the long-term interest and short-term interest extraction modules in chronological order. The brief process is shown in Figure 2.
(3)   Reward function: when designing the reward function, this paper uses the difference between the predicted score and the real score as the criterion to guide the optimization direction of the intelligent body. The specific design approach is as follows:
  (5) $$\begin{array}{c} \text{Reward}=e^{-\left(abs\left(\text{pre}\_\text{score}-\text{real}\_\text{score}\right)\right)}\text{,} \end{array}$$

where pre-score indicates the predicted score, real_score indicates the real score, and abs indicates that the absolute value sign is taken. The reward function can be interpreted as follows: the larger the gap between the predicted score and the real score, the smaller the reward obtained by the intelligence, and the smaller the gap the larger the reward obtained.

In this paper, the performance of the algorithm is observed mainly through the trend of the rewards obtained by the intelligences to observe whether the algorithm eventually converges. In testing the convergence of the algorithm, because the test results of a single user are contingent and do not reflect the overall performance of the algorithm, this paper collects the rewards obtained by the intelligences of each record of each user during the test and reflects the convergence of the algorithm by calculating the mean value of the collected data. Thus, the final rewards used for testing take the form of

(6) $$\begin{array}{c} \text{Ave}\_\text{reward}=\frac{\sum_{i}\sum_{j}r_{ij}}{N}\text{.} \end{array}$$

The effectiveness of the algorithm is tested using the root mean square error (RMSE) and the mean absolute error (MAE), which are common test metrics for rating classification algorithms. The RMSE and MAE are expressed as

(7) $$\begin{array}{c} \text{RMSE}=\sqrt{\frac{1}{m}\overset{m}{\underset{i=1}{\sum }}{\left(y_{i}-{\hat{y}}_{i}\right)}^{2}}\text{,}\\ MAE=\frac{1}{m}\overset{m}{\underset{i=1}{\sum }}\left|y_{i}-{\hat{y}}_{i}\right|\text{.} \end{array}$$

### 4.1. Experimental Results and Analysis

#### 4.1.1. Overall Performance Comparison

Therefore, after the analysis of Tables 4–6, the performance of the deep reinforcement learning algorithm based on the extraction of public service infrastructure. The specific results are given in Tables 4–6.

#### 4.1.2. Analysis of Algorithm Convergence

This part of the experiment mainly collects the Reward value Reward that the intelligent body can obtain after each prediction recommendation score when the algorithm is tested, as well as the RMSE and MAE values that can be obtained for each round of prediction, and analyzes the convergence of the algorithm by observing the trend of the values of these evaluation indexes. Also, in order to evaluate the convergence of the algorithm as a whole, this paper analyzes the algorithm by observing the trend of the average return Ave_Reward in each round.  Figure 3 shows the trend graph of the Ave_Reward values of the DDPG-LA algorithm and the combined algorithm of each module with increasing number of training sessions on both data sets.

From Figure 3, it can be seen that the overall results of all algorithms tested on the dataset are better.

#### 4.1.3. Comparative Analysis of Discount Factor *γ*

In the experimental process to get the best experimental results, this paper tries various different discount factor values and visualizes the effect of each discount factor through the final results. And by comparing the height of the curves, it is found that the height of the curve changes with the value of *γ* from small to large, and the trend of this correlation is shown in Figure 4.

The Total_Ave_Reward value represents the average of the average Reward for each round of testing at different *γ* values, i.e.,

(8) $$\begin{array}{c} \frac{1}{n}\overset{n}{\underset{i=1}{\sum }}\text{Ave}\_{\text{Reward}}_{i}\text{,} \end{array}$$

where *n* denotes the number of test rounds. Figure 4 shows that different discount factors have an effect on the final convergence of the algorithm and are positively correlated.

## 5. Conclusion

The needs of social development, the support of national policies, and the support of information technology have created a very favorable environment for the development of smart cities and become a strong impetus for the smooth development of smart cities. In practice, construction planners tend to pay too much attention to the input of technology and its effect to meet expectations, while ignoring the inner needs of thousands of city dwellers, that is, ignoring the essence of “service.” Before making a decision, a comprehensive and large-scale survey should be conducted to identify the needs of the residents, and on this basis, a plan should be designed to make the city a livable place that is recognized by the people through artificial intelligence-based methods, rather than operating according to the criteria that the decision makers have in mind. The concept of smart cities continues to rise in popularity, with more and more voices participating in the discussion, and it is normal for misconceptions and deviations to occur, but as decision makers and builders, it is important to clearly understand where the original intention of developing smart cities lies, to think about its essence and connotation in an environment where the heat remains high, and to make decisions that are truly relevant.

## Figures and Tables

**Figure 1:** Schematic diagram of deep reinforcement learning-based recommendation system.

**Figure 2:** Sketch of state generation.

**Figure 3:** Ave_Reward trend graph.

**Figure 4:** Trend of total_ave_reward value for different values of *γ*.

**Algorithm 1:** SCR algorithm.

**Table 1:** Descriptive statistics of each variable.

Variable name	Sample size	Mean value	Standard error	Min	Maximum value
PE	155	16.187	2.35	12.13	18.99
SC	155	3.197	0.65	1.32	4.51
MHC	155	8.933	2.06	5.39	18.21
HC	155	545.798	445.21	42.12	2293.69
PC	155	0.699	0.55	0.28	3.28
SS	155	28.798	10.05	8.31	65.21
DI	155	0.245	0.21	0	1.00
DO	155	0.205	0.23	0	1.00
GDP	155	0.279	0.19	0	1.00
FDI	155	0.152	0.21	0	1.00
INF	155	0.556	0.23	0	1.00
PS	155	0.387	0.28	0	1.00

**Table 2:** Basic regression analysis.

Public services	Model	DI		DO		Fixed effects	Time effect	Control variables	*N*	*R* ^2^
Public education	1	−4.029	(2.268)	0.153	(1.325)	√	×	×	155	0.049
	2	−5.055	(0.569)	−1.195	(1.387)	√	√	×	155	0.103
	3	−5.348	(2.446)	−0.352	(1.396)	√	×	√	154	0.069
	4	−5.987	(2.568)	−0.935	(1.558)	√	√	√	154	0.129

Social security	5	−1.921	(1.281)	−0.093	(0.265)	√	×	×	155	0.061
	6	−1.202	(1.178)	0.510	(0.389)	√	√	×	155	0.151
	7	−0.857	(0.935)	1.754	(0.558)	√	×	√	154	0.269
	8	−0.635	(0.976)	1.727	(0.597)	√	√	√	154	0.289

Health care	9	7.267	(3.825)	0.907	(0.955)	√	×	×	155	0.051
	10	5.854	(3.789)	−2.062	(1.263)	√	√	×	155	0.188
	11	6.395	(4.223)	−1.358	(1.989)	√	×	√	154	0.071
	12	6.236	(3.512)	−1.598	(1.539)	√	√	√	154	0.223

Housing	13	485.002	(386.698)	1694.899	(230.699)	√	×	×	155	0.739
	14	101.899	(435.698)	1357.400	(268.000)	√	√	×	155	0.798
	15	62.001	(435.199)	555.200	(286.000)	√	×	√	154	0.855
	16	25.031	(424.899)	599.100	(283.000)	√	√	√	154	0.859

Public culture	17	0.212	(0.285)	0.868	(0.145)	√	×	×	155	0.738
	18	−0.115	(0.283)	0.539	(0.142)	√	√	×	155	0.798
	19	0.035	(0.302)	0.435	(0.161)	√	×	√	154	0.855
	20	−0.062	(0.289)	0.469	(0.129)	√	√	√	154	0.865

Social services	21	−4.359	(19.798)	8.779	(10.188)	√	×	×	155	0.659
	22	6.987	(25.268)	9.899	(13.872)	√	√	×	155	0.789
	23	−25.599	(18.982)	23.835	(12.599)	√	×	√	154	0.755
	24	−16.029	(19.525)	15.001	(14.232)	√	√	√	154	0.132

**Table 3:** Heterogeneity regression results.

Public services	Category	DI		DO		*N*	*R* ^2^
	*A*	−3.321	(3.159)	0.122	(2.155)	55	0.299
	*B*	−11.563	(4.712)	−1.456	(3.652)	50	0.367
	*C*	−5.698	(6.312)	−10.799	(5.235)	49	0.451
	East	−2.156	(3.038)	−0.195	(2.659)	60	0.191
	Central	−10.179	(9.068)	−8.985	(7.334)	45	0.412
	West	−10132	(5.556)	−3.178	(2.894)	49	0.468

Social security	*A*	−2.049	(0.953)	0.522	(0.688)	55	0.293
	*B*	2.036	(1.478)	1.623	(0.915)	50	0.595
	*C*	−6.599	(3.523)	2.998	(0.820)	49	0.645
	East	−0.152	(1.132)	1.293	(0.652)	60	0.265
	Central	0.323	(2.598)	2.187	(0.126)	45	0.371
	West	−5.236	(2.239)	1.789	(1.569)	49	0.525

Health care	*A*	9.156	(1.650)	−5.123	(1.002)	55	0.253
	*B*	2.968	(5.469)	−1.489	(2.006)	50	0.372
	*C*	9.367	(19.185)	−11.321	(15.865)	49	0.521
	East	7.152	(3.339)	−2.789	(3.422)	60	0.820
	Central	−0.705	(5.525)	−13.569	(4.335)	45	0.453
	West	16.598	(12.635)	−3.155	(5.985)	49	0.203

Housing	*A*	44.003	(486.200)	−563.651	(280.400)	55	0.429
	*B*	−39.598	(345.900)	−116.987	(230.400)	50	0.719
	*C*	539.251	(398.200)	68.487	(328.200)	49	0.235
	East	666.798	(575.600)	356.000	(515.300)	60	0.968
	Central	1298.362	(420.400)	522.400	(288.600)	45	0.897
	West	−122.000	(415.200)	470.000	(265.400)	49	0.921

Public culture	*A*	0.036	(0.449)	0.022	(0.142)	55	0.893
	*B*	0.061	(0.272)	−0.055	(0.188)	50	0.926
	*C*	−0.698	(0.345)	−2.179	(0.455)	49	0.906
	East	0.309	(0.455)	0.279	(0.195)	60	0.896
	Central	0–0.049	(0.355)	−0.035	(0.295)	45	0.897
	West	−0.255	(0.519)	−0.263	(0.196)	49	0.793

Social services	*A*	7.186	(25.325)	1.059	(12.725)	55	0.879
	*B*	−37.269	(23.805)	34.100	(17.655)	50	0.931
	*C*	187.399	(117.825)	46.168	(77.165)	49	0.756
	East	−15.598	(21.155)	16.239	(10285)	60	0.425
	Central	18.459	(36.825)	−49.179	(30.958)	45	0.498
	West	91.897	(135.895)	58.235	(35.889)	49	0.620

**Table 4:** Comparison of experimental results.

Algorithm	Dataset 1		Dataset 2	
	Ave_RMSE	Ave_MAE	Ave_RMSE	Ave_MAE
SCR	0.3992	0.2288	0.2776	0.1115
DDPG + RLSTM	0.4580	0.2616	0.5222	0.4085
DDPG + LETM	0.5892	0.4659	0.5568	0.4439
DDPG + *T*_self_attention	0.5762	0.4025	0.4486	0.2826
DDPG + self_attention	0.5965	0.44259	0.5356	0.3636
DDPG + RLSTM + self_attention	0.4025	0.2419	0.8552	0.1818
DDPG + LSTM + *T*_self_attention	0.4036	0.2358	0.6658	0.2860
DDPG + LSTM + self_attention	0.4478	0.2886	0.6829	0.3259
KNNBasic	0.9228	0.7476	0.6658	0.4201
KNNWithMeans	0.9320	0.7386	0.9886	0.7325
KNNBasicline	0.8958	0.7066	0.9335	0.7136
SVD	0.8830	0.6856	0.9258	0.7022
SVD++	0.8622	0.9728	09225	0.7268
NMF	0.9216	0.7352	0.9680	0.7698

**Table 5:** Boost values of SCR and module combination algorithm on Ave_RMSE.

		KNNBasic	KNNWithMeans	KNNBasicline	SVD	SVD++	NMF
*D*1	SCR	0.5225	0.5288	0.4958	0.4873	0.4562	0.5216
	DDPG + RLSTM	0.4848	0.4820	0.4562	0.7592	0.4212	0.4879
	DDPG + LETM	0.3258	0.3352	0.3568	0.2252	0.3210	0.3215
	DDPG + T_self-attention	0.3465	0.3525	0.2365	0.6582	0.3242	0.4521
	DDPG + self-attention	0.3288	0.3355	0.1598	0.7830	0.2826	0.4663
	DDPG + RLSTM + self-attention	0.5220	0.5268	0.2256	0.1259	0.2789	0.3221
	DDPG + LSTM + *T*_self-attention	0.5122	0.5255	0.3558	0.2525	0.2345	0.5124
	DDPG + LSTM + self-attention	0.4680	0.4820	0.7035	0.3251	0.2325	0.5110

*D*2	SCR	0.7535	0.7078	0.6524	0.3256	0.2451	0.3654
	DDPG + RLSTM	0.4568	0.4258	0.4125	0.2564	0.3214	0.3219
	DDPG + LETM	0.4256	0.3865	0.3254	0.6871	0.4004	0.2598
	DDPG + T_self-attention	0.5325	0.5226	0.4687	0.3252	0.6587	0.3987
	DDPG + self-attention	0.4452	0.4226	0.1036	0.2520	0.2335	0.4210
	DDPG + RLSTM + self-attention	0.1569	0.1298	0.7255	0.3210	0.5632	0.2113
	DDPG + LSTM + *T*_self-attention	0.3250	0.2826	0.3652	0.1020	0.1235	0.1558
	DDPG + LSTM + self-attention	0.3055	0.2678	0.5529	0.2325	0.2558	0.2864

**Table 6:** Lift values of SCR and module combination algorithm on Ave_MAE.

		KNNBasic	KNNWithMeans	KNNBasicline	SVD	SVD++	NMF
*D*1	SCR	0.4886	0.8098	0.4776	0.4568	0.4432	0.4862
	DDPG + RLSTM	0.4650	0.4886	0.4446	0.4250	0.4112	0.4620
	DDPG + LETM	0.2525	0.2692	0.2456	0.2268	0.2032	0.2556
	DDPG + *T*_self-attention	0.3256	0.3365	0.3005	0.2826	0.2688	0.3228
	DDPG + self-attention	0.3001	0.3225	0.2687	0.2642	0.2545	0.2788
	DDPG + RLSTM + self-attention	0.4865	0.5065	0.4856	0.4652	0.2459	0.4825
	DDPG + LSTM + *T*_self-attention	0.4935	0.5225	0.4826	0.4515	0.4340	0.4896
	DDPG + LSTM + self-attention	0.4358	0.4488	0.4268	0.4525	0.4368	0.4456

*D*2	SCR	0.6612	0.6325	0.6258	0.3898	0.3958	0.6548
	DDPG + RLSTM	0.3632	0.3342	0.3445	0.6352	0.6098	0.3588
	DDPG + LETM	0.3330	0.3095	0.3026	0.3280	0.3112	0.3128
	DDPG + *T*_self-attention	0.5220	0.4882	0.4682	0.3002	0.2001	0.4858
	DDPG + self-attention	0.488	0.3952	0.3846	0.2966	0.1987	0.3987
	DDPG + RLSTM + self-attention	0.0044	−0.0196	−0.0352	−0.0320	−0.4680	−0.0106
	DDPG + LSTM + *T*_self-attention	0.2090	0.1849	0.1568	0.1822	0.1562	0.1952
	DDPG + LSTM + self-attention	0.1826	0.1658	0.1423	0.1552	0.1283	0.1658

## Data Availability

The experimental data used to support the findings of this study are available from the corresponding author upon request.
